The article "The Diagnostic Evaluation of the SINEH Cardiopulmonary Triage Scale and the Emergency Severity Index in the Emergency Department: A Comparative Study" was published in 2024. Journal: Emerg Med Int.

# The Diagnostic Evaluation of the SINEH Cardiopulmonary Triage Scale and the Emergency Severity Index in the Emergency Department: A Comparative Study

**DOI:** 10.1155/2024/3018777

**Published:** 2024-03-22

**Authors:** Mahbobeh VatanKhah, Javad Malekzadeh, Mohammad-Davood Sharifi, Amir Mirhaghi

**Affiliations:** ^1^Intensive Care Nursing, Student Research Committee, Nursing and Midwifery School, Mashhad University of Medical Sciences, Mashhad, Iran; ^2^Department of Prehospital Emergency Care, School of Nursing and Midwifery, Mashhad University of Medical Sciences, Mashhad, Iran; ^3^Department of Emergency Medicine, Faculty of Medicine, Mashhad University of Medical Sciences, Mashhad, Iran; ^4^Nursing and Midwifery Care Research Center, School of Nursing and Midwifery, Mashhad University of Medical Sciences, Mashhad, Iran

## Abstract

**Introduction:**

The diagnostic evaluation of the emergency severity index (ESI) in the triage of patients with cardiopulmonary complaints has a high sensitivity but a low specificity in the emergency department (ED). Therefore, triage scales with more accurate diagnostic evaluation are required. As a result, accuracy of the SINEH triage scale (SinTS) and the ESI was compared to compare mistriage of critically ill patients with cardiopulmonary complaints.

**Methods:**

This descriptive, analytical and cross-sectional study was conducted between December 2022 and April 2023. In this study, two nurses independently examined each patient using two triage scales. The admission unit and length of hospital stay were also recorded. The outcome was classified as high-risk admission (cardiac care unit and intensive care unit) and low-risk admission (internal unit or discharge from the ED). Undertriage and overtiage were defined as high-risk admission with triage level 3 and 4 and low-risk admission with triage level 1 or 2, respectively. A panel of experts evaluated content validity of SinTS and kappa designating agreement on relevance reported. The inter-rater reliability of two scales was also reported.

**Results:**

Finally, the study included 145 patients. The average age of the patients studied was 61.35 years. SinTS has a total mistriage of 29.63%, with 4.13% being undertriage and 25.5% being overtriage. In ESI, the total mistriage is 66.8%, with 1.3% being undertriage and 65.5% being overtriage. The undertriage of the two scales did not differ significantly by admission unit (*p*=0.26), but the overtriage of the two methods did (*p*=0.001). The sensitivity, specificity, and accuracy of SinTS were 86.3%, 63.37%, and 72.27%, respectively, while those of ESI were 95.4%, 5.94%, and 32.79%, respectively.

**Conclusion:**

SINEH triage scale has achieved the optimal accuracy in recognizing the acuity of the patients with chest pain and dyspnea by using SpO_2_, pressure of end-tidal carbon dioxide, troponin I, and peak expiratory flow. When triaging patients with chest pain and dyspnea, SinTS may exhibit a higher level of accuracy compared to ESI. More research is needed to improve accuracy of triage scales in patient with cardiopulmonary complaints.

The article "The Diagnostic Evaluation of the SINEH Cardiopulmonary Triage Scale and the Emergency Severity Index in the Emergency Department: A Comparative Study" was published in 2024. Journal: Emerg Med Int.

## 1. Introduction

Prioritization of care and treatment for patients in the hospital is defined as triage [1]. Mistriage is a major concern in triage of critically ill patients. The most common diagnostic tools in triage scales are vital signs, but their sensitivity and specificity are limited [2]. As the clinical expertise of triage nurses varies, triage scales were developed to provide a more comprehensive approach to triaging the patients. There are two types of triage scales in terms of clinical complaint domain: general triage scales and specialized or informative triage scales. The Emergency Severity Index (ESI) triage is a general scale designed for all clinical complaints that is heavily reliant on the vital signs and clinical expertise of the triage nurse [3]. The ESI scale is reliable because it is simple and easy to use. The triage nurses' clinical expertise allows them to identify high-risk situations and the probable used resources [4]. Because of the significant role of triage nurse, the mistriage of ESI is reported in a wide range in literature [5–7]. Overtriage is the most common types of mistriage in the ESI, the cause of which can be traced back to the level-2 criteria, where the “high-risk situation” can be interpreted differently [3]. On the other hand, the patient's allocation to the level 2 is indirectly related to vital signs, which can lead to overtriage too. This mistriage is especially noticeable in case of chest pain or dyspnea complaint. In addition to the foregoing, the definition of used resources for cardiac or pulmonary complaints usually includes more than two scores even in noncritical situation and this also causes mistriage. Therefore, we decided to see if a triage scale specifically designed for cardiac and pulmonary complaints could significantly reduce mistriage in ESI triage performance. The SINEH cardiopulmonary triage scale (SinTS) is a four-level specialized scale designed for triaging patients with complaints of chest pain and dyspnea. In Persian, SINEH means “chest.” This scale evolved from the five triage scales developed since 2016 [2, 5–8]. This scale was structured using criteria such as peripheral oxygen saturation (SpO_2_), pressure of end-tidal carbon dioxide (PetCO_2_), respiratory rate (RR), blood pressure (BP), high sensitive troponin I (hs-cTnI), peak expiratory flow (PEF), and other evidence-based risk criteria. The sum of these criteria can lead to patients being examined based on physiological and quantitative criteria, and patient triage is less reliant on the clinical expertise of the triage nurse. As a result, the purpose of this study was to compare the diagnostic evaluation of the SinTS and ESI.

The article "The Diagnostic Evaluation of the SINEH Cardiopulmonary Triage Scale and the Emergency Severity Index in the Emergency Department: A Comparative Study" was published in 2024. Journal: Emerg Med Int.

## 2. Method

This descriptive, analytical, and cross-sectional study was carried out between December 2022 and April 2023 to compare the diagnostic evaluation of SinTS and ESI. In this study, each patient was triaged using SinTS and ESI by two nurses. The research was carried out in the ED of Imam Reza Hospital in Mashad, Khorasan Razavi. Every month, this ED sees 10,000 patients with various complaints. This hospital has both specialized and general units. The fourth version of the 5-level ESI triage system is used in this ED [9]. The ESI is a simple to use, five-level triage algorithm that priorities emergency patients by evaluating both patient acuity and resource needs. Initially, the triage nurse assesses only the acuity level. If a patient does not meet high acuity level criteria (ESI level 1 or 2), the triage nurse then evaluates expected resource needs to help determine a triage level (ESI level 3, 4, or 5) [9]. In this ED, level 1 and 2 patients are transferred to the acute section, level 3 patients to the examination section, and level 4 and 5 patients to the outpatient section in the ED.

### 2.1. Ethical Considerations

The Mashhad University of Medical Sciences Ethics Committee approved this study (IR.MUMS.NURSE.REC.1401.042). The patients provided informed consent. The patients were assigned to triage level using the department's routine method (ESI). At the same time, another nurse allocated triage level based on SinTS. As a result, each patient was triaged by two scales. Safety protocol was implemented to prevent the transmission of infection through the respiratory assessment devices.

### 2.2. Design

The study included patients who complained of chest pain and dyspnea. Patients over the age of 18 years with no history of recent trauma were also included. Exclusion criteria included transfer to other hospital in less than 6 hours, incomplete file information, a diagnosis other than cardiopulmonary disease, and intolerance to capnography or peak flowmeter. Each patient was independently triaged by the ED nurse (who performed ESI) and the researcher nurse (who performed SinTS). Both researchers had 10 years of working in the ED and 2 years of triage experience. The two nurses were kept blind toward triage parameters of the opposing method. Finally, the patient was referred to the ED based on ESI triage.

The article "The Diagnostic Evaluation of the SINEH Cardiopulmonary Triage Scale and the Emergency Severity Index in the Emergency Department: A Comparative Study" was published in 2024. Journal: Emerg Med Int.

### 2.3. SinTS

The researcher first takes the patient's vital signs (RR and SpO_2_) and then uses the capnometer device to measure the PetCO_2_. If these parameters are normal, the patient's systolic BP (SBP) is also measured; if any of them are abnormal (SpO_2_ ≤ 80% or RR ≥ 32 bpm or PetCO_2_·≤ 23 mm hg or SBP ≤ 90 mm hg), the patient is assigned to the level 1; otherwise, level 2 is assigned. In the following step, if any of the criteria (92% > SpO_2_ > 80% or 28 mm hg > PetCO_2_ > 23 mm hg) had an abnormal value, they are assigned to the level 2, and if they were normal, they are referred to decision box C. If the criteria (SpO_2_ ≥ 92% and PetCO_2_ ≥ 28 mm hg) were normal and the patient had high-risk cardiac and pulmonary criteria, she/he is assigned to the level 3 based on decision box C, provided that Box C-1 is not fulfilled. Chest pain patients with positive troponin or dyspneic patients with high-risk peak flowmeter value (PEF ≤ 50% of expected) or all patients with unbearable pain are assigned to the level 2. Finally, if the patient does not meet the high-risk criteria, she/he will be placed in level 4 (Figure 1).

### 2.4. ESI

The triage nurse in Imam Reza Hospital's Edalatian Emergency Department classifies patients based on the ESI triage (fourth version) during the assessment. Patients are classified into five levels. Levels 4 and 5 are considered as level 4 in this study because they are both referred to the outpatient section.

### 2.5. Outcomes

The admission unit included intensive care unit (ICU), cardiac care unit (CCU), internal unit (IU), and discharge from the ED. In addition, the length of hospital stay (hours) for each patient was calculated.

### 2.6. Content Validity of the Instrument

The researcher-made triage scale used in this study was compiled by reviewing the most recent studies on high-risk signs and symptoms related to the short-term mortality in patients with chest pain or dyspnea complaints (Figure 1). The items were organized into triage levels, and the corresponding level was chosen based on the risk ratio for each sign and symptom introduced in the studies. This instrument was presented to a group of experts in order to calculate the content validity index (CVI). The Scale-CVI was calculated using the kappa designing agreement on relevance [10]. The Scale-CVI was 0.847.

The capnography device (BCI® Capno check® plus) was used. Device measures RR, SpO_2_, and PetCO_2_. Disposable cannula was used to assess respiratory criteria. Accuracy of PetCO_2_ measurement is 2 mm hg. Test-retest reliability of capnography was 0.990. High sensitive troponin rapid kit, in a few minutes, with a cut-off point of 1 ng/L determines troponin I (cTnI) based on a drop of blood from the patient's finger. The sensitivity and specificity of the rapid troponin kit exceeded 97%. The peak flowmeter device (Rosemax) had an accuracy of 20 liters per minute (LPM). Test-retest reliability of PEF was 0.999. Protective filter was used to prevent transmission of respiratory disease.

The article "The Diagnostic Evaluation of the SINEH Cardiopulmonary Triage Scale and the Emergency Severity Index in the Emergency Department: A Comparative Study" was published in 2024. Journal: Emerg Med Int.

### 2.7. Reliability

Two nurses assessed the reliability of SinTS and ESI for 20 patients. The inter-rater agreement was used to assess reliability, and the kappa coefficient of agreement for SinTS and ESI was 0.688 and 0.605, respectively.

### 2.8. Sample Size

A post hoc power analysis was performed based on the odd ratio of admission unit (SinTS 3.4; ESI 0.49), and it showed study power of 0.97 and 0.94, respectively.

### 2.9. Statistical Analysis

After collecting and coding the data, analysis was performed using SPSS software version 22 in this study. To describe the characteristics of the study sample, descriptive statistics such as relative frequency distribution, mean and standard deviation, and minimum and maximum values were reported. To compare variables between SinTS and ESI triage levels, ANOVA and Wilcoxon were used. Chi-square and Fisher's exact were used to examine the independence of association between nominal variables. The reliability was evaluated using the inter-rater assessment method (kappa). Polit and Beck's content validity index was used to assess the content validity of the researcher's scale. Because the confidence coefficient of 95% (*α* = 5%) was used, a significant difference was reported in cases where *P* < 0.05. Patients with high-risk outcomes (CCU and ICU) were considered positives for the diagnostic evaluation of patients in both scales, separately in a 2 × 2 table, while IU admission and discharge from the ED were considered negatives, and level 1 and 2 were also considered positive, in contrast to level 3 and 4 which were negative. Pearson coefficient was used to assess test-retest reliability of PEF and PetCO_2_.

## 3. Results

The study included 165 patients. Nine patients left the ED against medical advice and 11 patients did not want to participate in the study. Finally, the study included 145 patients. The mean age of patients was 61.35 ± 14.64 years. Female made up 53.1% of the sample size. Ambulances transported 21% of patients to the ED. Triage took 2.38 ± 0.6 minutes (mins) and lasted between 1 and 5 mins. Sixty percent of the patients reported chest pain, and 40% reported dyspnea. Patients were diagnosed acute coronary syndrome (ACS) 50%, chronic obstructive pulmonary disease (COPD) 12%, and other diagnoses 38%. Patients who discharged from the ED were 47.6%, 22% were admitted to the IU, and 30.4% were admitted to critical units (CCU and ICU) (Table 1).

The article "The Diagnostic Evaluation of the SINEH Cardiopulmonary Triage Scale and the Emergency Severity Index in the Emergency Department: A Comparative Study" was published in 2024. Journal: Emerg Med Int.

### 3.1. Mistriage

The total mistriage of the SinTS is 29.63%, with 4.13% undertriage and 25.5% overtriage based on the outcome of the admission unit (admission to the CCU and ICU vs. discharge from the ED and admission to the IU). In ESI, the total mistriage is 66.8%, with 1.3% being undertriage and 65.5% being overtriage. The undertriage of the two scales did not differ significantly based on admission unit (*p*=0.26), but the overtriage of the two scales did (*p*=0.001).

### 3.2. Diagnostic Evaluation

Based on the admission unit and hospital stay, the diagnostic evaluation of the SinTS and ESI is described (Table 2).

Table 3 explains the mean and standard deviation of SpO_2_ and PetCO_2_ for each triage level. It is worth noting that 21% of the 89 subjects tested positive for cTnI and all of them had normal vital signs. Only two PEF of 110 and 130 LPM were performed.  Table 4 shows a description of vital signs based on admission unit.

## 4. Discussion

This triage scale has been developed from the five previous triage scales used since 2016, including the cardiac triage scale, heart failure triage scale (HFTS), ESI plus PEF, ESI plus cTnI, and ESI plus PetCO_2_ [2, 5–8]. Today, it is necessary to use informative or specialty scales for triage of critically ill patients and refining previous triage scales with the recent advancement of research. Furthermore, due to patient overcrowding, it is inevitable to use specialized scales rather than general scales designed for all complaints, just as they switched from 3-level to 5-level triage scales, aiming for more precise triage scales. SinTS has created a favorable accuracy for patient triage, particularly for patients with high-risk complaints such as chest pain and dyspnea, by using specific criteria of SpO_2_ and PEF for COPD patients, PetCO_2_ for HF patients, and cTnI for MI patients. These complaints are most closely related to mortality, and they account for roughly half of all presenting complaints in the ED, which should be paid attention as much as possible.

Based on admission unit outcome, the total mistriage is 29.63% in SinTS and 66.8% in ESI. Mistriage of ESI was found to be 32.2% in a study of 5 million ED patients, with 28.9% being overtriage and 3.3% being undertriage [11]. Because our study only included high-risk patients with complaints of chest pain and dyspnea, a mistriage of 66.8% for ESI was reported in comparison to Saxs' study. When triaging patients with chest pain complaint, nurses typically evaluate them as a high-risk situation and assign them to triage level 2. When we consider that nearly half of all ED visits are chest pain, we can see that, in the absence of quantitative criteria for triaging patients with chest pain, triage nurses are cautious to avoid mistriage [12]. The main risk that nurses are concerned about is myocardial infarction (MI). In clinical symptoms of MI, chest pain has a high sensitivity but a low specificity, so the triage nurse assigns any patient with chest pain or discomfort to level 2 to avoid mistriage [13]. As a result of the poor diagnostic value of chest pain, adding quantitative criteria such as the rapid troponin test can reduce significantly mistriage. Using a cTnI in ESI to triage patients with low-risk chest pain reduced overtriage from 88% to 6% [5]. Another noteworthy issue is that the patients with MI in this study (19 patients) had positive troponin, despite having normal vital signs, and this situation increases the possibility of undertriage if the nurse underestimates patient's chest pain and fails to recognize the high-risk situation. Furthermore, approximately 33% of patients with a MI do not have chest pain [13]. As a result of using the rapid troponin test in triage, there is less mistriage for patients with chest pain, and the triage nurse can assign a patient with chest pain who has normal vital signs and a negative troponin to a less acuity level safely.

The article "The Diagnostic Evaluation of the SINEH Cardiopulmonary Triage Scale and the Emergency Severity Index in the Emergency Department: A Comparative Study" was published in 2024. Journal: Emerg Med Int.

HF patients make up a considerable proportion of ED patients, who frequently present with dyspnea. In the triage of patients with dyspnea, SpO_2_ is usually regarded as the most important factor in determining the acuity of the condition. Because measuring RR is difficult for nurses [14] and it can be influenced by the sympathetic nervous system, anxiety, and even recent short-term activities, its measurement in triage can be associated with false positive results (undertriage). The time-consuming measurement of the RR, combined with the lack of RR measurement tool in triage, forces the triage nurse to rely on SpO_2_ measurement extensively, which is quick and easy to obtain. Patients with HF (killip Class 1 or 2) on the other hand, usually have normal or near-normal SpO_2_ [2, 7, 15]. Only when they reach killip class 3, their SpO_2_ significantly decrease to 85% [15]. Patients hospitalized in critical units (ICU and CCU) had a mean SpO_2_ of 91.86% (mild hypoxemia) in this study, which is not considered high-risk criteria, based on SpO_2_ and is thus consistent with previous studies (Table 4) [2, 7]. As a result, it is critical to note that SpO_2_ does not have sufficient sensitivity (65% for SpO_2_ < 93%) to determine the acuity of HF patients, implying that a significant portion of patients is ignored and undertriage occurs. Even when the triage nurse is cautious, this problem causes 10% undertriage in these patients [7]. Undertriage can be aggravated when it is discovered that frequent visits to the ED by these patients can reduce the sensitivity of nurses and may assign them to less acuity level, resulting in undertriage of up to 20.5% [7]. PetCO_2_ is more effective than SpO_2_ [2] in reducing mistriage in HF patients because it detects a drop in cardiac output and a decrease in pulmonary blood flow with a sensitivity and specificity of 76.6% and 75%, respectively [16]. PetCO_2_ explains 28.1% and left ventricular ejection fraction explains 67.5% of occurrence of major cardiovascular events, and both play a role in predicting the acuity of HF patients [17]. As a result, the use of PetCO_2_ for monitoring the acuity of HF patients is recommended [16, 17]. Adding PetCO_2_ to ESI reduced mistriage in HF patients from 41% to 10% [2]. This study's findings are also consistent with the preceding because the mean PetCO_2_ for patients admitted to the CCU and ICU was 31.31 mm Hg, which differed from the values for patients admitted to other units (Table 4). This suggests that PetCO_2_ may be a more effective measure than SpO_2_ in determining the acuity of HF patients. The PetCO_2_ cutoff point for predicting severity of HF patients has been varied from 32.1 to 32.2 mm Hg in literature [16, 17]. However, because the triage of patients with short outcomes was considered in this study, cut-off points of 23 and 28 mm Hg were used for level 1 and 2 in SinTS, respectively. More research is required to determine the best cut-off point for predicting short outcomes in patients with HF. There is vertical validity for PetCO_2_ in SinTS in this study, but because this criterion was not measured in ESI, there is no significant difference between the ESI triage levels in this regard, and the ESI criteria could not detect significant difference in HF patients (Table 3).

The article "The Diagnostic Evaluation of the SINEH Cardiopulmonary Triage Scale and the Emergency Severity Index in the Emergency Department: A Comparative Study" was published in 2024. Journal: Emerg Med Int.

Patients with COPD exacerbation are another subgroup of patients who visit ED with dyspnea. SpO_2_ criteria in these patients may also be associated with some degree of mistriage. First, SpO_2_ may temporarily be overestimated by increasing RR [6]. Furthermore, in COPD patients, the difference between SpO_2_ and SaO_2_ has been reported to be up to 3.39%, implying that SpO_2_ is 3.39% higher than SaO_2_, and this mistriage reaches up to 8% during moderate hypoxia, resulting in normoxia (false negative results) [18]. In this line, SpO_2_ has a sensitivity and specificity of 84.6% and 87.5% for the diagnosis of respiratory failure, respectively. As a result, SpO_2_ criteria in COPD patients should be interpreted with caution, and this issue should be considered on triage scales to reduce undertriage. In this study, only 12% of patients presented with a complaint of dyspnea were diagnosed as COPD exacerbation, and nearly all of them were admitted to the IU after the relative stability of their general condition; thus, the mean SpO_2_ in the IU was 86.65%, and the mean RR was 29.78 per minute. Because the patients were admitted to the IU with improved respiratory condition after receiving oxygen, bronchodilator, and antibiotic drugs in the ED, they did not need to be admitted to the ICU (Table 4). As a result, in SinTS, the SpO_2_ criterion was set at less than 80% for level 1 and 92% for level 2, ensuring that only patients in extremely high-risk situations are assigned to level 1 and hospitalized in an ICU if necessary. In contrast, defining the need for “life-saving intervention” in ESI can result in a overtriage. Because the urgent need for oxygen therapy can be a reason for the triage nurse to assign patients with COPD exacerbation to the triage level 1, then these patients quickly experience a relative improvement in their general condition and are finally admitted to the IU, and there is no need for them to be admitted to ICU, which endangers the ESI validity. In SinTS, patients with SpO_2_ less than 80% were assigned to level 1, so that only very high-risk patients were admitted. PEF was used when triage nurse was uncertain about triage of COPD patients with normal SpO_2_. Only two cases of PEF of 110 and 130 lpm were performed in this study as an aid in diagnosing high-risk COPD patients. A PEF reading of 120.2 + 36.7 lpm has been linked to an increased likelihood of COPD patients being admitted to the hospital [19]. By incorporating PEF into ESI, mistriage was reduced from 42.85% to 2.85% [6]. In this study, maximum PEF less than 50% of the expected was considered as a criterion for level 2, and PEF between 50% and 80% of the expected was considered as a criterion for level 3. More research is needed to determine the appropriate PEF cut-off point and its role in prioritizing patients in the triage of patients with COPD exacerbation.

Based on the admission unit outcome, the sensitivity and specificity of SinTS were 86.3% and 63.37%, respectively (Table 2). The outcome of admission unit (ICU and CCU) was strongly related to the hospital stay >12 hours. Both gold standards produced similar diagnostic evaluation results for critically ill patents (level 1 and 2). The sensitivity and specificity ESI were 95.4% and 5.94%, respectively. This demonstrates that the overtriage (false positive) in ESI was significant, at 65.5%. The reasons for this overtriage have previously been discussed, and they are primarily due to the high-risk features of patients with cardiac and respiratory complaints, as well as the poor diagnostic evaluation of cardiopulmonary signs and symptoms [2, 5, 6, 11]. Because of this issue, the accuracy of ESI is 32.79% and the accuracy of SinTS is 72.27%. SinTS produced comparable results to other triage scales that used informative triage scales to determine the severity of patients' conditions. The sensitivity and specificity of the FTS, which includes an ECG, were 61% and 76%, respectively [20].

The article "The Diagnostic Evaluation of the SINEH Cardiopulmonary Triage Scale and the Emergency Severity Index in the Emergency Department: A Comparative Study" was published in 2024. Journal: Emerg Med Int.

A study on the diagnostic evaluation of four scales of ESI, MTS, Australian Triage Scale (ATS), and Canadian Triage and Acuity Scale (CTAS) found that their sensitivity and specificity are similar, with sensitivity ranging between 91% and 93% and specificity ranging between 34% and 41% [21]. This suggests that, in the absence of diagnostic aids, triage scales for triaging patients with chest pain result in high sensitivity and low specificity in order to avoid mistriage as much as possible. This study also compared the results with the FTS, which included an ECG, and discovered that when the ECG is used in triage, the sensitivity decreases to 71% and the specificity increases to 68%, and false positive results or overtriage is reduced. This increase in specificity was caused by an increase in the triage nurse's ability to reduce undertriage (false negative). The overall accuracy of all of these scales, however, has been reported to be between 64% and 69% in Dechamps' study [21]. Increasing specificity and reducing false negatives through the use of ECG may increase the false positive error and reduce the sensitivity of the scale. As a result, more research is needed to determine diagnostic criteria of ECG in triage. In this regard, adding a capnometer to ESI could increase specificity in the triage of HF patients from 42.6% to 60% [2]. Sensitivity, specificity, and accuracy of SinTS demonstrated 86.3%, 63.37%, and 72.27%, respectively, which is higher than Dechamps's study because SinTS used rapid troponin to diagnose high-risk ACS patients, which has a higher diagnostic value than ECG. The results of diagnostic evaluation of ESI are consistent with previous findings of high sensitivity and low specificity in the literature. However, the sensitivity of ESI in this study was 95.4%, which was higher than previous studies, because the patients in this study were all patients with high-risk complaints of chest pain or dyspnea, and 22% of them were hospitalized in CCU and ICU, and thus this overtriage rate is to be expected in the absence of diagnostic aids (Table 1). Other recent studies have found high sensitivity but low specificity for other scales. A study on the diagnostic evaluation of the MTS for the triage of patients with ACS revealed a sensitivity of 70–80% and a specificity of 59% [22]. A recent study for the MTS found that it had a sensitivity and specificity of 45.7% and 84.8% in diagnosing critically ill patients with chest pain, respectively, and an accuracy of 81.9% [23]. The scale's reliance on the clinical expertise of the triage nurse has increased heterogeneity between studies and expanded the scope of the scale's diagnostic evaluation results [22, 24, 25]. In fact, it is possible to conclude that triage scales for determining the acuity of patients with chest pain complaints have high sensitivity and overtriage (false positive) to avoid ignoring patients with ACS. This is because clinical signs and symptoms of ACS, such as retrosternal pain, have high sensitivity but low specificity, forcing the triage nurse to assign patients to level 1 or 2, which may result in substantial overtriage rate. On the other hand, the introduction of diagnostic tools such as ECG reduces undertriage and increases specificity, allowing more patients to be assigned to the level 3 or 4; however, some of the sensitivity may decrease, resulting in overtriage. As a result, cTnI, which has higher sensitivity and specificity than ECG, can play a more accurate role in diagnosing critically ill patients without compromising triage accuracy.

The article "The Diagnostic Evaluation of the SINEH Cardiopulmonary Triage Scale and the Emergency Severity Index in the Emergency Department: A Comparative Study" was published in 2024. Journal: Emerg Med Int.

The gold standard of admission unit was used in this study. In triage studies, gold standards include death, hospitalization in ICU and CCU, high-risk events such as MI, used resources, length of hospital stay, invasive interventions such as cardiopulmonary resuscitation, and so on. The admission unit had a strong relationship with the length of hospital stay in this study, because the length of hospitalization is usually a function of the relevant admission unit. Patients may be admitted to the unit for reasons other than the acuity of their condition; for example, some hospitals have guidelines that allow patients in stable condition to be admitted to the CCU for elective diagnostic angiography. Therefore, local guidelines may bias diagnostic evaluation results, reduce the accuracy of triage scales, and be considered as research limitations. However, in general, this gold standard is reliable and has been used in numerous studies and there was a significant correlation between admission unit and length of hospital stay.

Another limitation is the triage nurse's clinical expertise. The clinical expertise of the triage nurse may be one of the most important of heterogeneity factors between studies, expanding the range of results between similar studies. In this study, nurses with more than ten years of experience in the ED were recruited for triage so that they had the sufficient competence for triaging patients. However, when compared to other scales, clinical expertise of triage nurses had little effect on SinTS. The allocation of patients to level 1 and 2 is based primarily on physiological and quantitative criteria. However, in ESI, decision-making of level 1 and 2 is largely subjective and based on the clinical expertise of the triage nurse, which studies have linked them to overtriage [3]. The values of SpO_2_ in two scales in Table 3 show that there is horizontal validity in both scales, and level 1 has the lowest SpO_2_ of 82.55% and 81.55% in SinTS and ESI, respectively, and it differs significantly from other levels. These findings showed that triage nurses had sufficient adherence to triage scales.

The article "The Diagnostic Evaluation of the SINEH Cardiopulmonary Triage Scale and the Emergency Severity Index in the Emergency Department: A Comparative Study" was published in 2024. Journal: Emerg Med Int.

SinTS employs a capnometer, rapid troponin kit, and peak flowmeter, which may not be available in all triage departments, limiting its use. However, with the overcrowding of patients in EDs, it is unavoidable to adopt more precise methods for patient entry into EDs and to increase patient safety. This scale can be used for hospital triage in an acceptable time range of 1 to 5 minutes. The troponin kit produces preliminary results in a matter of minutes. In a few seconds, capnometry can determine the RR and ETCO_2_. Peak flowmetery takes less than a minute. All of these measurements are not required in all patients, and level 1 or 2 patients can be identified in a few seconds with abnormal SpO_2_ or PetCO_2_, while level 3 patients can wait longer due to the general stability of vital signs. An important point to remember is that evidence-based decision-making by triage nurses can improve patient safety in the ED and prevent mistriage, which leads to the use of emergency resources and fatigue among department nurses and endangers patients' safety.

Despite the fact that the power in this study is greater than 0.8, in order to reproduce the same results, this study must be conducted with a larger sample size and in multiple centers. Given that the majority of the study criteria are set quantitatively and the role of the triage nurse's clinical expertise is limited, it is expected that these results can be replicated in other studies. It is also worth noting that the research on the cut-off point of SpO_2_ criteria, PetCO_2_, cTnI, PEF, and RR may require further investigation and refining. Patients suffering from anxiety attacks, for example, may have a high RR and low PetCO_2_ and be assigned to level 1, despite the fact that they are not in immediate danger, resulting in an overtriage. These patients quickly achieve general stability and are discharged without hospitalization after a brief treatment in the ED, which can reduce the sensitivity of the triage scale. To prevent this kind of mistriage, full attention must be paid to patient's history and the role of previous medical disease.

The article "The Diagnostic Evaluation of the SINEH Cardiopulmonary Triage Scale and the Emergency Severity Index in the Emergency Department: A Comparative Study" was published in 2024. Journal: Emerg Med Int.

## 5. Conclusion

The SinTS has achieved the optimal accuracy in determining the acuity of patients with chest pain and dyspnea by using SpO_2_, PetCO_2_, cTnI, and PEF. This scale has acceptable horizontal validity in addition to good vertical validity because patients with chest pain and dyspnea are both triaged using the same scale. Because of the reliance of SinTS on advanced vital signs and physiological findings related to MI, HF, and COPD, the role of clinical expertise of nurses in patient triage has been diminished. As a result, in the triage of patients with chest pain and dyspnea, SinTS may be more accurate than ESI. More research is needed to improve triage scales in this subgroup of patient.

## Figures and Tables

**Figure 1:** SINEH triage scale (SinTS) for patients with cardiopulmonary complaints (Ver.1). Details 1: unbearable chest pain: it is a chest pain that the patient cannot stand to perform a hs-cTnI due to the severity of the pain. High-risk cardiac profile: unstable angina, unstable angina (moderate to severe pain; prolonged and increasing; at rest), history of heart disease, diabetes. Mellitus, age >50 years, pacemaker, left ventricular ejection fraction <35%, dysrhythmia, critical changes in other vital signs. High-risk pulmonary profile: maximum expiratory flow (PEF) between 50% and 80%, history of lung disease, history of heart failure or liver disease, smoking, age >70 years, hospitalization history >4 times in the last year, CRP >10 mg/dl, leukopenia, use of secondary muscles of respiration, fever. PetCO_2_: pressure of end-tidal CO_2_, hs-cTnI: high sensitivity cardiac troponin I, and PEF: peak expiratory flow.

**Table 1:** Patient distribution based on admission unit and level of triage.

	CCU and ICU admission *n* = 69 (%)		Internal unit admission *n* = 32 (%)		Discharged from ED *n* = 44 (%)		Total *n* = 145 (%)	
	SinTS	ESI	SinTS	ESI	SinTS	ESI	SinTS	ESI
Level I	15 (10.3)	11 (7.6)	16 (11)	11 (7.6)	7 (4.8)	5 (3.4)	38 (26.2)	5 (7.2)
Level II	23 (15.9)	31 (21.4)	7 (4.8)	20 (13.8)	7 (4.8)	59 (40.7)	37 (25.5)	59 (85.5)
Level III	5 (3.4)	1 (0.7)	9 (6.2)	1 (0.7)	45 (31)	2 (1.4)	59 (40.7)	2 (2.9)
Level IV	1 (0.7)	1 (0.7)	0 (0)	0 (0)	10 (6.9)	3 (2.1)	11 (7.6)	3 (4.3)
	Chi-square = 8.08, *df* = 1, *p*=0.045		Chi-square = 5.02, *df* = 1, *p*=0.025		Chi-square = 7.46, *df* = 1, *p*=0.006		Chi-square = 5.4, *df* = 1, *p*=0.037	

The article "The Diagnostic Evaluation of the SINEH Cardiopulmonary Triage Scale and the Emergency Severity Index in the Emergency Department: A Comparative Study" was published in 2024. Journal: Emerg Med Int.

**Table 2:** Diagnostic evaluation of triage scales based on admission unit and hospital stay.

Triage scale	Based on admission in CCU and ICU vs IU and discharged from ED		Based on length of hospital stay (>12 hours vs <12 hours)	
	SinTS	ESI	SinTS	ESI
Sensitivity	0.86 (72.65–94.83)	95.4 (84.5–99.4)	76.25 (65.42–85.05)	96.25 (89.43–99.22)
Specificity	63.37 (53.19–72.73)	5.94 (2.21–12.48)	78.46 (66.51–87.69)	7.69 (2.54–17.05)
PPV	50.26 (38.47–62.02)	30.31 (22.75–38.74)	55.43 (43.5–66.92)	26.81 (19.61–35.05)
NPV	91.56 (82.43–96.87)	75.31 (35.19–96.92)	93.39 (80.96–96.13)	85.38 (45.06–99.41)
Accuracy	72.27 (62.12–77.56)	32.79 (25.23–41.07)	77.89 (70.25–84.35)	30.72 (23.33–38.91)

**Table 3:** Mean of SpO_2_ and PetCO_2_ criteria for each level of triage scales.

	SpO_2_ (%)		PetCO_2_ (mm Hg)	
	SinTS	ESI	SinTS	ESI
Level I	82.55 ± 13.96	81.55 ± 15.89	28.65 ± 10.86	34.55 ± 8.49
Level II	93.91 ± 4.23	94.7 ± 5.05	34.89 ± 5.46	32.93 ± 7.1
Level III	96.59 ± 2.21	93.5 ± 3.1	35.03 ± 3.98	37.25 ± 3.86
Level IV	97.54 ± 1.69	97.75 ± 1.7	36.9 ± 3.28	37.00 ± 1.82
	*H* = 49.38, *df* = 3, *P*=0.001	*H* = 21.37, *df* = 3, *P*=0.001	*H* = 22.01, *df* = 3, *P*=0.001	*H* = 4.06, *df* = 3, *P*=0.225

**Table 4:** Mean and SD of vital signs criteria based on admission unit.

	SpO_2_ (%)	PetCO_2_ (mm Hg)	RR (min)	SBP (mm Hg)	DBP (mm Hg)	PR (bpm)
Discharged from ED	95.18 ± 4.61	34.28 ± 5.57	22.98 ± 7.6	153.11 ± 29.72	91.78 ± 21.25	88.46 ± 20.84
Internal unit	86.65 ± 12.97	34.65 ± 9.26	29.78 ± 10.17	143.68 ± 36.16	86.0 ± 22.12	97.84 ± 20.15
CCU and ICU	91.86 ± 10.78	31.31 ± 7.7	24.81 ± 8.05	141.5 ± 30.96	85.02 ± 20.27	84.45 ± 18.21
Total	92.30 ± 9.59	33.46 ± 7.28	25.04 ± 8.72	147.51 ± 31.84	88.45 ± 21.25	89.31 ± 20.38
	*H* = 12.33, *df* = 2, *P*=0.002	*H* = 7.73, *df* = 2, *P*=0.021	*H* = 11.97, *df* = 2, *P*=0.003	*F* = 2.11, *df* = 2, *P*=0.124	*H* = 3.46, *df* = 2, *P*=0.177	*F* = 4.3, *df* = 2, *P*=0.015

## Data Availability

Data will be shared upon reasonable request to the corresponding author with permission from Mashhad University of Medical Sciences..
